The article "Marine Macroalgae Display Bioreductant Efficacy for Fabricating Metallic Nanoparticles: Intra/Extracellular Mechanism and Potential Biomedical Applications" was published in 2021. Journal: Bioinorg Chem Appl.

# Marine Macroalgae Display Bioreductant Efficacy for Fabricating Metallic Nanoparticles: Intra/Extracellular Mechanism and Potential Biomedical Applications

**DOI:** 10.1155/2021/5985377

**Published:** 2021-11-27

**Authors:** Sabiha Mahmood Ansari, Quaiser Saquib, Valeria De Matteis, Hend Awad Alwathnani, Sulaiman Ali Alharbi, Abdulaziz Ali Al-Khedhairy

**Affiliations:** ^1^Botany & Microbiology Department, College of Science, King Saud University, P.O. Box 2455, Riyadh 11451, Saudi Arabia; ^2^Zoology Department, College of Science, King Saud University, P.O. Box 2455, Riyadh 11451, Saudi Arabia; ^3^Department of Mathematics and Physics “E. De Giorgi”, University of Salento, Via per Arnesano, 73100 Lecce, Italy

## Abstract

The application of hazardous chemicals during nanoparticle (NP) synthesis has raised alarming concerns pertaining to their biocompatibility and equally to the environmental harmlessness. In the recent decade, nanotechnological research has made a gigantic shift in order to include the natural resources to produce biogenic NPs. Within this approach, researchers have utilized marine resources such as macroalgae and microalgae, land plants, bacteria, fungi, yeast, actinomycetes, and viruses to synthesize NPs. Marine macroalgae (brown, red, and green) are rich in polysaccharides including alginates, fucose-containing sulfated polysaccharides (FCSPs), galactans, agars or carrageenans, semicrystalline cellulose, ulvans, and hemicelluloses. Phytochemicals are abundant in phenols, tannins, alkaloids, terpenoids, and vitamins. However, microorganisms have an abundance of active compounds ranging from sugar molecules, enzymes, canonical membrane proteins, reductase enzymes (NADH and NADPH), membrane proteins to many more. The prime reason for using the aforesaid entities in the metallic NPs synthesis is based on their intrinsic properties to act as bioreductants, having the capability to reduce and cap the metal ions into stabilized NPs. Several green NPs have been verified for their biocompatibility in human cells. Bioactive constituents from the above resources have been found on the green metallic NPs, which has demonstrated their efficacies as prospective antibiotics and anti-cancer agents against a range of human pathogens and cancer cells. Moreover, these NPs can be characterized for the size, shapes, functional groups, surface properties, porosity, hydrodynamic stability, and surface charge using different characterization techniques. The novelty and originality of this review is that we provide recent research compilations on green synthesis of NPs by marine macroalgae and other biological sources (plant, bacteria, fungi, actinomycetes, yeast, and virus). Besides, we elaborated on the detailed intra- and extracellular mechanisms of NPs synthesis by marine macroalgae. The application of green NPs as anti-bacterial, anti-cancer, and popular methods of NPs characterization techniques has also been critically reviewed.

## 1. Introduction

The production of materials in the size range of 1–100 nm is the core concept of “nanotechnology” [1]. Over the last few decades, nanoparticles (NPs) have been intensively studied owing to their unique physiochemical properties. Characteristic changes at nanoscale allow the NPs to be used in different applications viz chemical, electronic, electrical, mechanical, magnetic, thermal, dielectric, optical, and biological [2, 3]. Consequently, NPs are contemplated as building blocks for the next generation of technology. Nano research across the globe has been intensified to synthesize NPs of definite shapes and sizes. Several physical and chemical processes including lithography, sol-gel synthesis, aerosol technology, chemical reduction, and laser ablation can generate varying types of NPs [4, 5], to name a few nanodisks, nanowires, nanocubes, and nanorods [6–9]. Nonetheless, the methods adopted for NPs synthesis employ toxic chemicals as reducing agent and organic solvents or nonbiodegradable as stabilizing agents. Though physical and chemical methods are more popular for NPs synthesis, the use of toxic compounds limits their wide applications. Chemicals used in NPs synthesis are highly reactive, posing serious threats to the environment and equally not safe for humans. Above all, the upscale production of NPs using chemical methods is quite expensive and requires time-consuming processes. It is evidenced that metallic NPs can induce toxicity, either directly or indirectly by interacting with cells, and release toxic metal ions [10]. Hence, to reduce the toxicity, green processes of capping and nucleation of metallic NPs have been done, which enhanced their stability and dispersion and simultaneously augmented their anti-cancer efficacies [10]. The biological process has been preferred as a safe and eco-friendly approach for the major production of NPs [11]. Microorganisms, marine organisms, algae, microfluids, and plant extracts have exhibited their metal-reducing properties. Therefore, new prospects for the biogenesis of NPs have been opened [12–17]. The green approach popularly includes Tollens reaction [18]. In addition, green approach has successfully used polysaccharides [19], mixed-valence polyoxometalates [20], and irradiation methods [21]. Ideally, the green synthesis of NPs utilizes the biological extracts of a living microorganism, which acts as a reducing and capping agent. Combinations of polysaccharides, vitamins, amino acids, enzymes, and proteins in the biological fluid help reduce the metal ions into their corresponding NPs.

For ages, humans are relying on nature for basic needs, and plenty of bioactive agents originally developed from natural sources. Oceans cover around 70% of the Earth's surface, with tremendous variations in the biodiversity [22]. In view of the diversity and high endemism in marine biota, research on marine organisms offers unique advantages. Marine natural products from different sources exhibited diversification in chemical structures, as well as their biological activities. One indispensable component of the marine ecosystem is “macroalgae,” which utilizes sunlight to produce carbohydrates from carbon dioxide and water. Apart from balancing the marine ecosystem, scientists have found that macroalgae are important sources of protein, iodine, vitamins, minerals, and polyphenols [23, 24]. For several years, macroalgae and their extracts have been utilized as a fresh source of bioactive compounds with immense medicinal potential in the pharmaceutical industry [25]. Macroalgae were reported containing compounds including anti-bacterial and anti-tumor activities [26, 27]. Such benefits prompted the nanotech industries to use macroalgae as a biological source for the green synthesis of NPs. In spite of the fact, there is paucity of information on the mechanistic aspect of NPs synthesis using algae. Also, research done on green synthesis of NPs using marine macroalgae is disseminated. Hence, the above information gaps have motivated us to provide a source of comprehensive information on up-to-date research done on the green synthesis of NPs using marine macroalgae. We also encouraged to discuss the mechanism of NPs synthesis by the marine macroalgae along with a discussion of their cellular compositions, which is rarely reported anywhere. We carefully reviewed the current knowledge on the green synthesis of metallic NPs by marine macroalgae and microalgae and the related mechanism of intra- and extracellular mode of NPs synthesis. In addition, we also studied the biogenic production of metallic NPs using plants, bacteria, viruses, fungi, and yeast. Lastly, we presented some frequently used techniques of NPs characterizations and application of biogenic metallic NPs as anti-cancer and anti-microbial entities.

## 2. What Are Nanoparticles (NPs)?

Nanotechnology is a novel branch of science, which blends the principles of biology and physical and chemical sciences that generate nano-sized particles harboring specific functions [28–31]. NPs are a kind of materials that typically range between 1 nm and 100 nm (Figure 1). Compared to the bulk material, NPs have unique physicochemical properties due to their high surface area to volume ratio. Reduced cohesive energy (especially the surface atoms at sharp corners and edges become very reactive) and a higher degree of curvature provide excellent properties to NPs to act as a catalyst for surface-sensitive reactions [32]. At the nanoscale, uneven distribution of electrons leads to magnetic properties in NPs [33]. NPs also demonstrated fluorescence/photoluminescence properties at nanoscale due to interband radiative transitions and also radiative decay of surface plasmons [34]. NPs can be engineered by different kinds of chemical substances. Organic dendrimers, semiconductor nanocrystals, carbon fullerenes, and carbon nanotubes are some of them [35]. However, NPs can be generated naturally via different environmental processes including weathering of rocks, forest fires, volcanic eruptions, soil erosions, explosion of clay minerals, and sandstorms [36]. At the nanoscale, NPs exhibit different sizes and shapes. Such remarkable characteristics bring revolution in different fields; thus, NPs have paved a way for novel fields in therapeutics, optoelectronics, drug discovery, diagnostic biological probes, catalysis, display instruments, biological sensors, and detection of environmental toxic metals or reagents [37–41]. Several types of NPs have been synthesized, including metallic and nonmetallic NPs such as gold, silver, palladium, platinum, zinc oxide, and titanium oxide NPs. These nanoobjects have been widely used owing to their excellent electronic, mechanical, optical, chemical, and magnetic properties [42–47].

## 3. Methods for the Synthesis of NPs

NPs can be synthesized by two fundamental approaches: the top-down and the bottom-up approaches (Figure 2). Within the top-down approach, NPs are generated by slicing the size of their bulk counterpart employing several physical and chemical methods [48]. The top-down approach can be achieved using the microfabrication techniques, where external tools are applied to precisely cut, mill, and change the material into a desired size and structure [33, 49]. Microfabrication techniques are of different types including laser ablation, etching, sputtering, mechanical milling, and electro-explosion [50–53]. Comparatively, within the bottom-up approach, NPs production involves the assembly of small entities together like atom by atom, molecule by molecule, and cluster by cluster. Hence, it is also referred to as “molecular nanotechnology” [54]. The nano-sized structures produced by the bottom-up approach cover several methods such as chemical reduction, plasma or frame spraying, sol-gel process, molecular condensation, supercritical fluid synthesis, laser pyrolysis, use of templates, chemical vapor deposition, and most significantly the green synthesis [55–63].

NPs generated using the abovementioned approaches have exhibited less defects, and they showed homogenous chemical compositions. However, the prime focus in these methods was to synthesize NPs of varying sizes with different chemical compositions, monodispersion, and specific morphologies [64, 65]. In both approaches (top-down and bottom-up), the NPs synthesis is achieved by kinetic processes, which help determine the size and shapes of NPs (Figure 2). The growth rate and energy of crystals are monitored by employing the surfactants and templates assisting to curtail the interfacial energy [33, 66]. While NPs synthesis, surfactants can be used as a capping agent to alter the surface morphology of NPs. Most commonly used surfactants include thioglycerol, sodium dodecyl sulfate, cetyl trimethyl ammonium bromide, polyvinylpyrrolidone, sodium hexametaphosphate, and mercaptoethanol [65]. In addition, the color change of the reaction solution also serves as a strong indicator of NPs synthesis.

## 4. Biological Materials for NPs Synthesis

Nowadays, biological entities are in high demand for NPs synthesis, as compared to chemical methods. A wide variety of marine and freshwater algae, plants, bacteria, actinomycetes, fungus, viruses, and yeast have been successfully utilized for NPs synthesis because they are eco-friendly and inexpensive; more often, they are called “nanofactories” (Figure 3). These living entities vary in their biochemical processing potential, which can be utilized for the synthesis of metallic oxide and metallic NPs.

In fact, it is true that all organisms are unable to synthesize the NPs, possibly due to the restrictions of certain enzymatic activities and intrinsic metabolic activities. Consequently, before commencing NPs synthesis, careful thought is needed on the selection of organisms. In fact, those biological creatures, which have greater heavy metal accumulative potential, have exhibited the best chance to synthesize metallic NPs [66–69]. In this context, the suitability of algae has been found on the top of their structure. A possible reason for metal bioaccumulation by algae is related to their cell wall complexity, which is known to be composed of mucilaginous polysaccharides and carboxyl groups [70]. Especially, the marine macroalgae growing in different conditions such as acidic, alkaline, hypersaline, and large range of temperature. It has been proven that these organisms act as a good source for the biosynthesis of NPs due to the presence of biologically important metabolites. On the other hand, plant materials are another source for the biological synthesis of NPs. The diverse chemical constituents present in plant extracts act as reducing and stabilizing or capping agents during NPs synthesis [45, 71–73]. The other facet of NPs synthesis using biological sources includes the use of microorganisms. Several factors such as light, pH of the medium, temperature, nutrients, mixing speed, and buffer strength all play an important role in the enzyme activity [63, 74]. Moreover, the biosynthesis of metallic NPs is considered an important technique of the green chemistry method that links nanotechnology and microbial biotechnology [75].

Scientists have also utilized macromolecules (DNA and proteins) and enzymes for the synthesis of biocompatible NPs. For example, double-stranded DNA (dsDNA) was adsorbed on lanthanide-doped NPs to produce biosensors that have the ability to cross the cell membrane and are regarded for their prospective use in bioimaging and DNA delivery [67]. With the use of chimeric DNA molecules, nanocrystals with multiple ligands have been developed that exhibit the propensity to target different addresses in the cells [68, 69]. Ag-dsDNA-GO nanocomposite exhibited significant anti-bacterial effects by decreasing the *Xanthomonas perforans* cell viability in tomato plants [70]. In the same line, bovine serum albumin (BSA) has been utilized as a template to create Mn-doped zinc sulfide quantum dots (ZnS QDs) exhibiting phosphorescence properties that can be implemented as a biosensor [71]. QDs functionalized with BSA, lysozyme, trypsin, hemoglobin, and transferrin were developed that were highly luminescent and proposed to be suitable for cancer cell imaging [72]. Gold nanoparticles synthesized from green reducing agents of proteins by in situ reduction method demonstrated their sensing capabilities for different proteins [73]. Au-NPs have been synthesized using catecholamines, and their applicability has been suggested in the biomedical and bioanalytical fields [74].

## 5. Chemical versus Biological Methods for NPs Synthesis: Advantages and Disadvantages

NPs can be synthesized via different chemical methods including but not limited to chemical reduction, electrochemical, chemical precipitation, and hydrothermal approaches. Most of these methods use synthesis in homogeneous liquids such as water or organic solvents. Catalytic reduction method and flame spray pyrolysis are some of the other methods of NPs synthesis in a gaseous environment. Sol-gel and microemulsion methods are also used for the synthesis of NPs via the chemical method. Major advantages associated with chemical methods of NPs synthesis are that they are simple, have control over the size of NPs, and are cost-effective. In spite of the benefits, major disadvantages of chemical methods are the presence of impurities, high temperature, costly equipment, and use of toxic and hazardous chemicals that are non-eco-friendly and restrict their biomedical applications [75].

Green synthesis of NPs has manifold advantages in terms of cost, eco-friendly, and is biocompatible. Above all, this process does not require stabilizers due to the presence of cellular capping and stabilizing agents [76]. The surface of green synthesized NPs has the ability to adsorb biomolecules when they contact complex biological fluids. Consequently, they lead to the formation of the corona, thereby allowing their interaction with biological systems. The corona layers provide an auxiliary advantage over the naked biological NPs [77]. Medicinal plants and marine-based sources contain abundant metabolites exhibiting excellent pharmacological properties. The use of such sources for NPs synthesis allows the attachment of metabolites on the synthesized NPs, which can enhance their efficacies to be used in different applications [76, 78, 79]. Concerning the steps and time required in NPs synthesis, the biological approach needs fewer steps, as compared to chemical methods [36]. The chemically synthesized NPs must need an external attachment of the functional group for getting biological activity, while biologically generated NPs do not need such attachments [36]. Biocompatibility, like reduced metal cytotoxicity, is one of the core issues for the application of NPs in biomedical settings. NPs produced by biological routes are usually free from toxic contamination of by-products, which is typically found in the chemically synthesized NPs, thus limiting their prospective use in the biomedical sector [36]. Apart from that, biological routes can give undesired biological molecules, as can be cytogenic or teratogenic molecules depending on the natural source. Hence, before expanding its application in miscellaneous fields, it is always advisable to check in vitro toxicity before the use of NPs, even it is coming from biological routes. Additionally, biologically synthesized NPs have limitations including less control on size and shape, involvement of unspecified cell organelles, less output of NPs to be commercialized, and separation of NPs from the reaction mixture.

## 6. Green Synthesis of NPs

Nature has provided a plethora of nano- and microlength inorganic materials, which have the potential to generate a relatively novel and unexplored areas of research [1]. Despite the tremendous benefits that NPs own, the physical and chemical methods involve hazardous chemicals [4, 5, 80]. Consequently, there is high demand for the development of a safe and environment-friendly procedures for producing NPs, which do not require the exploitation of toxic chemicals. Metal NPs production via chemical or physical procedures is not gracious due to the involvement of reducing agents. These chemicals are highly reactive and toxic in nature; hence, not safe for human consumption or to the environment, and they are quite expensive for upscale production. It has been confirmed that metallic or bare NPs can induce toxicity by directly interacting with cells or indirectly by releasing the toxic metal ions. Consequently, to scale down the toxicological effects, researchers tend to cap or nucleate the bare NPs, which has shown dispersion, promising stability, and enhanced killing of cancer cells [10]. Green synthesis of NPs can be achieved by using biological sources; nowadays, algae is a popular choice owing to its higher ability to uptake metals, cheaper, uniquely structured, macroscopic, and environmentally effective [39, 41, 81, 82]. The benefit associated with the use of biological materials for the synthesis of NPs is that the toxic chemicals produced during the NPs synthesis can be easily degraded with the help of enzymes present in them [83, 84].

### 6.1. NPs Synthesis Using Algae

Prior to discussing the utilization of algae as a source of NPs synthesis, it is quite important to discuss here the concept of multicellularity that has been evolved at least 25 times during the evolutionary timeline of eukaryotes [85]. It is intriguing that only a handful of these multicellular lineages has been considered a complex multicellular organism. However, the complex multicellular has also been defined as the possession of a macroscopic body plan made of varying types of cells developed during the course of developmental programs during cell division and differentiation [86]. Under the umbrella of this definition, not only animals, land plants, and fungi are considered to demonstrate multicellularity; rather, three independently evolved lineages of macroalgae (brown, red, and green) are also included. The broad classification of algae can be done as brown algae (*Phaeophyta*), red algae (*Rhodophyta*), and green algae (*Chlorophyta*). However, based on the size, algae can be classified as macroalgae or microalgae. Macroalgae are seaweeds, multicellular, and larger in size. Comparatively, microalgae are single-celled and microscopic, which may be prokaryotic-like cyanobacteria (*Chloroxybacteria*), or it can be eukaryotic-like green algae (*Chlorophyta*). During the acquisition of multicellularity, the development of an adherent extracellular matrix (ECMs) was very crucial in macroalgae. ECMs permit the transition from cellular autonomy to cellular cooperation. ECMs are complicated supramolecular networks that provide flexibility and rigidity to the multicellular algal tissues. Apart from their structural role, ECMs regulate development and protect the cells from the outer medium, including protection against abiotic and biotic stresses. ECMs matrix is predominated with polysaccharides, which greatly vary among different phyla and lower taxonomic ranks. Marine algal ECMs possess sulfated polysaccharides [87]. The main cell wall (CW) components of brown macroalgae are the presence of anionic polysaccharides including alginates and fucose-containing sulfated polysaccharides (FCSPs). Red macroalgae ECMs contain sulfated galactans, agars, or carrageenans, which are galactose residues linked by alternating *β*-1,4 and *α*-1,3 glycosidic bonds. Comparatively, marine green macroalgae ECMs include four types of polysaccharides: semicrystalline cellulose, water-soluble ulvans, and two minor hemicelluloses: a xyloglucan and a glucuronan [88]. Marine brown, red, and green macroalgae have ample differences in their ECMs and intracellular biological contents; a comparative illustration is depicted in Figure 4. A comprehensive description of the ECMs constituents of brown, red, and green macroalgae is reported in the review of Kloareg et al. [89]. Marine macroalgae ECMs figures were adopted from the review of Kloareg et al. [89] and redrawn from the work of Deniaud-Bouët and coworkers [90], as well as updated from the following references for brown macroalgae [91–93], red macroalgae [94–96], and green macroalgae [97]. Algae are photoautotrophic and oxygenic in nature, which has the ability to bioaccumulate heavy metals. Such distinctive characteristic and their abundance as a raw material have attracted many researchers to look for a cleaner method for NPs synthesis [98]. We have found that a substantial amount of research on green synthesis of NPs employing marine macroalgae is either focused on gold or silver NPs production. Compared to other species of macroalgae, brown macroalgae have been exploited more due to their excellent property of metal uptake. Additionally, the cell wall of brown macroalgae is complex, containing plenty of mucilaginous polysaccharides and functional groups (carboxyl groups), which help in the uptake of heavy metals [99]. Polysaccharide secretion of fucoidans from the cell wall of marine brown macroalgae has exhibited plenty of application as anti-inflammatory, anti-viral, anti-coagulant, and anti-cancer agents. Fucoidans are also used in the cosmetic industries as anti-aging or whitening agents. Synthesis of gold NPs (AuNPs) from fucoidans has provided a fruitful alternative to the chemical methods [99]. Alginate, laminaran, and fucoidan are different polysaccharides isolated from marine brown macroalgae *Saccharina cichorioides* and *Fucus evanescens* have demonstrated their capabilities as reducing and stabilizing agents during the biogenic synthesis of silver NPs [100]. Very recently, on a different line, two brown macroalgae (*F. evanescens and S. cichorioides*) from Okhotsk Sea and Trinity Bay have been implemented for the synthesis of fucoidan-chitosan NPs. The authors have emphasized that the structure of fucoidan's and their molecular weight play a crucial role in NPs synthesis [101]. In this context, crude fucoidans obtained from *Sargassum muticum* by hot water extraction method (40–80°C) have demonstrated their ability to reduce gold and silver ions to gold NPs and silver NPs [102]. Fucoidan isolated from *Padina tetrastromatica* has demonstrated its reducing capability to successfully generate gold NPs [103]. Extracellular extract prepared from brown macroalgae (*S. muticum*) of Red Sea exhibited capping abilities for the formulation of biocompatible stable silver NPs [104]. Brown seaweed (*Sargassum crassifolium*) confirmed the reduction of iron precursors into magnetic iron oxide NPs [105]. *Sargassum wightii* has shown its capability of extracellular synthesis of gold, silver, and gold-silver-bimetallic NPs [13]. *S. wightii* has also exhibited extracellular rapid synthesis of gold NPs, ranging between the size of 8 and 12 nm [106]. Earlier, biomass derived from marine brown algae (*Fucus vesiculosus*) has displayed the biological reduction of metallic gold into gold NPs [107]. *Fucus gardeneri* collected from Kongsfjorden, Arctic Ocean, when extracted in hot water demonstrated its efficiency to reduce silver nitrate to silver NPs [108]. *Lobophora variegate* thallus was dried and extracted in hot water, exhibited metal-reducing properties by converting silver nitrate ions to analogous silver NPs [109]. *S. wightii* and *Valoniopsis pachynema* methanolic extracts prepared from the cold stripping method displayed the reduction of silver nitrate to silver NPs [110]. On a different side, a crude extract prepared from brown macroalgae (*Saragassum cervicorne*) has been implemented for the one-pot green synthesis of palladium nanocatalyst (PdNCs) in the size range 3.131 to 16.45 nm [111]. The dried powder of *Sargassum vulgare* extracted in hot water reduced the ferric chloride to iron oxide NPs ranging between 17.05 and 34.09 nm[112].

Researchers not only exploited the brown macroalgae; rather, some recent studies successfully availed the biogenic properties of red algae to green synthesize NPs. Extracellular extract of *Portieria hornemanni* prepared via heating approach has demonstrated its competence to reduce the silver nitrate solution to silver NPs [113]. Aqueous extract prepared by boiling the dried powder of red algae (*Gelidium corneum*) has been implemented to green synthesize silver NPs in the size range of 20–50 nm [114]. Red seaweed (*Chondrococcus hornemannii*) collected from the coastal area of Villoondi Theertham, India, processed for extracellular extract preparation through boiling method efficiently reduced the silver nitrate solution to silver NPs [115]. In previous work, extracellular synthesis of gold NPs has also been demonstrated by the marine red algae (*Kappaphycus alvarezii*) [116]. In the same context, another species of marine red algae (*Chondrus crispus*) showed its ability to green synthesize gold and silver NPs [98]. *Jania rubens*, a red macroalgae, has reduced the metallic salt (ferric chloride) to generate iron oxide NPs within the size of 22.22 to 33.33 nm [112]. On the other hand, green algae (*Tetraselmis kochinensis*) has also produced gold NPs from metallic gold precursors [117]. *Spirogyra insignis* is a green alga that has exhibited its ability of biogenic production of gold and silver NPs [98]. Aqueous extract prepared from marine green macroalgae (*Ulva fasciata*) demonstrated its reducing and stabilizing properties to synthesize 22.73 to 39.77 nm iron oxide NPs [112]. Within the same approach, extract prepared from green algae (*Dictyosphaerium* sp.) was recently used for the synthesis of gold NPs and novel gold nanoformulations loaded with diosgenin [118]. Researchers have also taken the advantage of unicellular *Chlorella vulgaris* dried biomass for the synthesis of tetrachloroaurate ions to generate algal-bound gold, which was subsequently reduced to gold NPs. The synthesized gold NPs exhibited diverse morphology including decahedral, tetrahedral, and icosahedral shapes, especially accumulated near the cell surfaces [119]. *C. vulgaris* extract has been exploited for the production of silver nanometre scale plates. This finding revealed the unique role of proteins, which acted as a reducing and stabilizing agent and also behaved as a shape-control modifier [120]. The dry biomass of *C. vulgaris* extracted in water added to palladium chloride solution resulted in the green synthesis of palladium NPs. The authors concluded that amide and polyol groups present in the extract were responsible for the formation of palladium NPs [121]. Several green algae (*Rhizoclonium fontinale*, *Ulva intestinalis*, *Chara zeylanica*, and *Pithophora oedogonia*) and cyanobacteria (*Phormidium valderianum*, *P. tenue*, and *Microcoleus chthonoplastes*) when exposed to hydrogen tetrachloroaurate solution produced intracellular gold NPs [122]. Furthermore, silver NPs have also been produced in the presence of light by marine *Chlorella salina*, *Chaetoceros calcitrans*, *Isochrysis galgana*, and *Tetraselmis gracilis* [123]. *P. oedogonia* (Mont.) Wittrock aqueous extract rapidly reduced the silver nitrate to silver NPs [124]. *C. vulgaris* has also been employed for the biosynthesis of silver NPs in the size range between 50 and 70 nm. The possible factors responsible for the green synthesis of silver NPs have been attributed to the functional groups such as amines, phenols, alcohols, ethers, and aromatic rings in the extract, which played an important role to reduce silver ions to silver NPs [125]. A green and facile biotemplating method has been deployed to fabricate monodisperse MnO/C microspheres for lithium-ion batteries using microalgae, resulting in a unique hollow porous structure in which MnO-NPs were tightly embedded into a porous carbon matrix that forms a penetrative shell [126]. *Hydrodictyon* sp. and *Oedogonium* sp. collected from freshwater of Indonesia reduced the silver nitrate to silver NPs [127]. Extracts prepared from green microalgae (*Botryococcus braunii*) have also reduced the copper acetate and silver nitrate into the stabilized form of copper NPs and silver NPs [128]. Alcohol extracts prepared from different green microalgae (*Lyngbya putealis*, *Chlorella* sp., *Oocystis* sp., and *Scenedesmus vacuolatus*) assisted the production of silver and silver chloride NPs. The biomolecules present in the extracts were liable for the capping and stabilization of NPs [129].

### 6.2. Mechanism of NPs Synthesis by Algae

Biogenic synthesis of NPs using algae can be achieved either intracellularly and extracellularly. In the case of intracellular synthesis, bioreduction of metal precursors present in the growth medium takes place in three phases (activation phase, growth phase, and termination phase). During the activation phase, metal ions move quickly towards the cell surface owing to the presence of amino, phosphate, carboxylic, thiol, and so on. In the growth phase, which is comparatively slow, metal ions cross the cell wall/cell membrane via cell transport systems. Once inside the cell, biochemical molecules (pigments, carbohydrates, anti-oxidants, phycobilins, oils, polyunsaturated fatty acids minerals, fats, chlorophylls, proteins, and phytochemicals) as well NADPH or NADPH-dependent reductase derived from metabolic processes (photosynthesis, nitrogen fixation, and respiration) aid on reducing the charge on metal ion to zero-valent state. Subsequently, in the growth phase, nucleated metal tends to join each other to form NPs that are of varying shapes and sizes and are thermodynamically stable. In the last (termination) phase, the final shape of NPs is acquired, which predominantly relies on factors such as pH, temperature, time, substrate concentration, static condition, and stirring control. A schematic representation exhibits the key intracellular reducing agents and processes that execute the reduction of metal precursor to generate intracellular NPs using algae (Figure 5).

On a different aspect, extracellular synthesis of NPs from algae can also be achieved via dual approaches. The first approach involves the extracellular matrix (ECMs) of algae. Metabolites, pigments, proteins, lipids, DNA, ions, enzymes, nonprotein RNA, sulfated polysaccharides, cellulose microfibril, and hemicellulose microfibril enzymes present in the ECMs effectively reduce metal ions at the surface (Figure 5). In the second approach, extraction of biological materials from algae biomass via boiling and nonboiling procedures can be done. Exudates of algal cells containing proteins (enzymes), DNA, RNA, metabolites, pigments, ions, hormones, lipids, anti-oxidants, reducing sugars, and polysaccharides effectively reduce the metal ions and precipitate them into corresponding NPs. The mechanism discussed in this section has been derived from the previously published reports on the green synthesis of NPs by algae and the structural composition of marine macroalgae [107, 130–137].

Extraction of biological materials from macroalgae allows the researchers to reduce metal precursors in a more controlled way *per se* the need of growing algae in laboratory conditions for NPs synthesis has been reduced. The extracellular approach of NPs synthesis is much more appropriate in terms of NPs purification or recovery. Nonetheless, some perquisites such as washing and blending of algal biomass are required [138]. Factors such as pH, temperature, concentration, and type of precursor metal, and substrate influence the shape, size, and agglomeration of NPs [135, 139]. High pH inhibits NPs agglomeration by the enhancement of reducing the power of functional groups [140, 141].

However, basic pH assists in the capping as well as stabilization of NPs via interaction with amine groups of surface-bound proteins as well as their residual amino acids [142]. Notwithstanding the fact, the type of algae also plays a crucial role in the dose-dependent production of NPs, either by extracellular or an intracellular method [135–137]. Illustration in Figure 6 displays the modified steps we have adopted in our laboratory for preparing the extracellular extract from marine macroalgae without a heating approach [143].

The extracellular solution was subjected to sonication to allow the extraction of water-soluble biological materials, which can be filtered and utilized for the reduction of metallic precursors via capping and stabilization to produce metallic NPs through the green approach. The extracellular mechanism of NPs synthesis involves the addition of the metal precursor (M^+^) with the aqueous extract of macroalgae, which contains several biological materials (DNA, RNA, proteins, enzymes, polyphenols, carbohydrates, fats, and vitamins) causing the reduction/nucleation (M^0^) of metal precursor. The reduced metal precursor will undergo aggregation, capping, and stabilization to generate metallic NPs (Figure 6). As mentioned above, time plays a crucial role in NPs synthesis. It has been found that extracellular synthesis of gold NPs using *Lyngbya majuscula* and *Spirulina subsalsa* extracts exhibited a time-dependent development of color, indicating the bioconversion of Au^3+^ to Au^0^ leading to the steady synthesis of gold NPs [140]. Similarly, green synthesis of fluorescent gold NPs has been accomplished using red alga (*Lemanea fluviatilis* (L.) C. Ag.) was found to be a function of reaction time, as confirmed by UV-visible spectra showing conspicuous SPR peak of gold at 530 nm [144]. The role of pH in extracellular NPs synthesis is evident with the use of brown algae (*F. vesiculosus*) for gold nanospheres formation. It was found that nanospheres formation takes place in two stages. In the first phase, no change in color was observed after the addition of metal precursors. However, in the second phase, a distinctive color change and reduction of gold ions and pH were observed, especially pH 7.0, which was found most optimal owing to the fact that both processes took place simultaneously [107].

### 6.3. NPs Synthesis by Plants

The application of plant materials for NPs synthesis has opened a different avenue in the field of NPs synthesis that coined a new terminology “phytonanotechnology.” This procedure is cost-effective, rapid, applicable, and eco-friendly. NPs produced using the aqueous extract of the plant have many advantages such as scalability, biocompatibility, and medical usage [145]. The phytochemical constituents in plant extracts (polyphenols, phenolic acids, alkaloids, sugars, terpenoids, and proteins) actively reduce and stabilize the metallic ions [146, 147]. Consequently, plant-based NPs synthesized using nontoxic nature of plants are best suited to meet the demand of NPs with varied applications in the environmental and medical areas. For instance, we have recently used *Aloe vera* bioactives to encapsulate the hematite nanoparticles (ALE-*α*-Fe_2_O_3_NPs) and adopted a cost-effective, one-step rapid method for the biofabrication of *Eucalyptus globulus* leaf extract (ELE) bioactives to produce functionalized CuONPs [148, 149]. We have also employed the leaf extract of *Cymbopogon citratus* for one-pot green synthesis of CuONPs and *Myristica fragrans* leaf ester capped-zinc oxide nanoparticles (ZnONPs) [150, 151]. MgO and MnO_2_ NPs were synthesized from the extract of medicinal plant (*Matricaria chamomilla*) significantly inhibited *Acidovorax oryzae*, causing bacterial brown stripe disease in rice [152]. Ag-NPs synthesized from different plant extracts (*A. absinthium, T. vulgaris,* and *H. lupulus*) have demonstrated their antioxidant properties and antimicrobial efficacies [153]. Ag-NPs synthesized using *Pelargonium endlicherianum* exhibited anti-microbial effects against a range of bacterial strains [154]. *Panax ginseng* used for the synthesis of gold and silver NPs has indicated the important role of medicinally important plants [155–157]. *Morus indica*, *Catharanthus roseus*, *Morus alba*, and *Cocos nucifera* extracts have also been used for the synthesis of Ag-NPs [31, 158–160]. *Rubus idaeus*, *Fragaria ananassa*, *Rubus fruticosus*, and red cabbage extracts have been exploited for the green synthesis of Au-NPs [161, 162]. It is intriguing that various plant parts (fruits, stems, roots, leaves, and their extracts) have been used for the synthesis of metal NPs [163]. However, the precise mechanism and the components responsible for plant-mediated synthetic NPs remain to be elucidated. It has been found that *Corallina officinalis* polyphenols (hydroxyl functional group) and the proteins carbonyl group assist in the stabilization of gold NPs [164]. Similarly, *Murraya koenigii* leaf extract has also been utilized for the synthesis and stabilization of gold and silver NPs [165]. However, the mechanism of NPs synthesis differs from plant to plant species [36]. In particular, specific components such as emodin, cyperoquinone, dietchequinone, and remirin found in xerophytes and mesophytic plants are useful for metal NPs synthesis. The presence of eugenol, the main terpenoid in *Cinnamomum zeylanicum*, has reported playing a crucial role in gold and silver NPs [76]. *C. zeylanicum* bark extract has been used for the synthesis of palladium NPs [166]. *Annona squamosa* peel extract has been reported reducing the palladium metal ions to palladium NPs in the range 75 to 85 nm [167]. While the leaf extract prepared from *Glycine max* demonstrated the formation of palladium NPs showed in the mean size of 15 nm [168]. In fact, *Coffea arabica* and *Camellia sinensis* extracts also demonstrated their ability to assist the synthesis of palladium NPs of different sizes (20 to 60 nm) [169]. Moreover, *Gardenia jasminoides* constituents (anti-oxidants, crocetin, crocins, and chlorogenic acid) act as both reducing and stabilizing agents to produce palladium NPs [170]. Plant extracts prepared from *Azadirachta indica*, *Ocimum sanctum*, and aqueous honey have been utilized for the synthesis of platinum NPs [171–173]. Palladium NPs (∼15 nm) were reported to be synthesized using the leaf extract of soybean and *Cinnamomum camphora* leaf [168, 174]. Plant extracts (*Aspalathus linearis*) and the fishtail fern, sago palm, rosy periwinkle, and holy basil have been utilized for the synthesis of ruthenium oxide NPs [175, 176]. The general scheme of plant-based green synthesis of NPs is shown in Figure 7.

### 6.4. NPs Synthesis by Bacteria

Amongst the organism-based NPs synthesis, microbes have been a popular choice for many researchers because they are cost-effective and easy to handle and culture. Microbes carry excellent metal accumulation potential, which assists the reduction of metal ions to their corresponding NPs by the presence of intracellular biomolecules and enzymes [178, 179]. Like algal biosynthesis of NPs, bacteria-mediated NPs synthesis can also be achieved by extracellular and intracellular methods. The intracellular mechanism of NPs production includes the transportation of positively charged metals through the negatively charged cell wall via diffusion; later, cell wall enzymes detoxify the metals into nontoxic metallic NPs [180]. In the extracellular mechanism, several enzymes viz nitrate reductase or hydroquinone synthesized by several fungi and prokaryotic organisms actively convert the metallic ions to metallic NPs. The detoxification mechanism by microorganisms involves metal binding or volatilization, and vacuole compartmentalization. During the metallic stress, microbes eliminate the toxic heavy metals via reduction and active efflux through the cell membrane and also accumulate them inside the cells. It has been evidenced that several cell transport systems (ion channels, ion pumps, endocytosis, lipid permeation, carrier-mediated transport, and lipid permeation) were involved in the influx of some heavy metals (nickel, silver, lead, and gold) [181]. In addition, some chelating agents such as siderophores mediate the absorption of metals and help them transport from the microbial cell [182]. Phytochelatins, which are derived from glutathione and metallothionein, a cysteine-rich protein, exhibited metal binding and detoxification properties in bacterial cells [183, 184]. Bacterial species that are frequently used for NPs synthesis include *Escherichia coli*, *Klebsiella pneumonia*, *Lactobacillus* sp., *Actinobacteria* sp., *Pseudomonas* sp.*, Bacillus cereu*s, and *Corynebacterium* sp. [1, 185–187]. *Pseudomonas stutzeri* exhibited silver NPs synthesis via NADH-dependent electron transfer, which finally reduces the silver ions to silver NPs [188]. Several marine bacteria such as *Cyanobacteria*, *Actinobacteria*, and *Proteobacteria* have also been used for the biosynthesis of metallic NPs [189]. The psychrotolerant bacteria isolated from the Antarctica region have also been utilized for the biosynthesis of semiconductor fluorescent NPs [190]. *Pseudomonas* sp. were able to biosynthesize cadmium sulfide-NPs [189]. *Rhodopseudomonas palustris* has also been found to produce intracellular cadmium sulfide NPs [191].

### 6.5. NPs Synthesis by Fungi and Yeast

Fungi have opened a straightforward and easy approach for the mycosynthesis of NPs. Besides the low cost and easy handling of fungi, their inherent properties of metal hyperaccumulation have made them a popular choice for the low-cost production of NPs [192]. Relative to bacteria, fungi have demonstrated a higher wall binding potential of metal salts with fungal biomass, resulting in a greater yield of NPs [192, 193]. Mainly, there are three mechanisms associated with the fungal biosynthesis of metal NPs that include electron shuttle quinones, nitrate reductase action, or the combination of both [192]. Several fungal enzymes (nitrate reductase, reductase, and NADPH-dependent reductases) produced from *Penicillium* and *Fusarium oxysporum* have played a significant role in NPs synthesis [194]. *F. oxysporum* when cultured with the aqueous extracts of TiF_6_^−2^ and Si_6_^−2^ successfully produced the titania and silica NPs [195]. In addition, marine multicellular fungi also demonstrated their ability to reduce the metals into the metallic NPs via extracellular and intracellular methods [196]. Gold and silver NPs have been reported to synthesize extracellularly by the use of cytosolic extracts and cell filtrate of *Candida albicans*, *Phoma glomerat*, *Penicillium fellutanum*, and *Penicillium chrysogenum* [197–201]. Platinum NPs have been synthesized extracellularly using the *F. oxysporum* ranging between 5 and 30 nm [202].

Yeast is another model for NPs synthesis by the green method. Its easy culturing method, rapid growth rate, and a large amount of enzyme production had given it an advantage over bacteria [203]. The extracellular extract of yeast cells (MKY3) has demonstrated their ability to reduce silver nitrate solution to very small-sized (2–5 nm) silver NPs [201]. *Schizosaccharomyces pombe* and *Candida glabrata* both have demonstrated their intracellular capabilities to produce cadmium sulfide NPs [204, 205]. Like bacteria and fungi, yeast cells under metal stress have developed the mechanism to detoxify their effects, usually by extracellular sequestration, chelation, biosorption, and bioprecipitation. Consequently, utilizing these mechanisms of yeast cells, one can generate stabilized NPs with different properties, sizes, and varying cellular locations [206]. It has been linked that *S. pombe* cells were able to produce cadmium sulfide-quantum dots at different growth phases [204, 207]. The regulation of growth and cellular activities of *Pichia jadinii* lead to the intracellular formation of different-sized gold NPs [208]. The influence of gold salt and biomass of *Yarrowia lipolytica* showed that both factors played a significant role in the formation of NPs with different sizes and morphology via extracellular and intracellular methods [146, 209].

### 6.6. NPs Synthesis by Actinomycetes and Viruses

Actinomycetes exhibit closer resemblance with fungi; although, differentiated as prokaryotes, can be easily modified genetically for the achievement of polydispersed and better sized NPs [210]. The properties of actinomycetes to produce antibiotics implicate them as a cleaner source for NPs production [211]. Actinomycetes have been found to generate different NPs via extracellular as well as intracellular methods. Extracellular mode is the most common pathway used by actinomycetes [212–214]. *Rhodococcus* sp. has reduced the metallic gold into nontoxic and monodispersed gold NPs, predominantly on its cell membrane and cell wall [212]. In the same context, several studies demonstrated the reduction of silver and gold ions to silver and gold NPs by the actinomycetes cell wall enzymes [215–218]. *Streptomyces capillispiralis*, an endophytic actinomycete, has shown its potential to generate nontoxic and eco-friendly copper NPs [219]. Actinomycetes isolated from soil have been reported reducing copper sulfate to copper oxide NPs [220]. Moreover, marine endophytic actinomycetes isolated from seaweeds have also demonstrated the reduction capabilities of copper sulfate to copper NPs [221].

In comparison to other microorganisms, the use of viruses for NPs synthesis is a quite different approach. Incubation of genetically modified M13 bacteriophage with zinc sulfide solution has resulted in the formation of zinc sulfide nanocrystals [222]. In the same line, the M13 bacteriophage is used for the orientation and nucleation of semiconductor nanowires [223]. The benefit of using viruses resides in the fact that they densely cover the surface of NP rings by capsid proteins, which result in the formation of a highly reactive surface that is capable of interacting with metallic ions [76]. On the other hand, tobacco mosaic virus (TMV) capsid protein acts like an attachment point for the deposition of materials [224–227]. The capsid protein of cowpea mosaic virus (CPMV) was found to electrostatically attach the palladium ions, which reduce and nucleate the metal ions to produce highly monodisperse metallic NPs [225]. Studies have confirmed that greater concentrations of TMV can give fewer free NPs; at the same time, TMV acted as a biotemplate that underwent metallization to form nanowires. Nanowires and nanotubes synthesized using viruses as a template were used in some earlier comparable studies [228, 229].

## 7. Techniques for the Characterization of NPs

Upon the successful synthesis of NPs, the next key target is to determine their sizes, distribution, shape, surface area, and surface morphologies. These parameters can be accomplished using varying spectroscopic and diffractographic techniques (Figure 8) [180, 230]. X-ray diffraction (XRD) measurement can quantify the diffraction patterns of NPs, which can be compared with the standard crystallographic database such as JCPDS to get structural information. Overall, XRD analysis can generate diverse information on the crystalline size, orientation and phases, purity, and geometry [230]. Scanning electron microscope (SEM) provides information about the dispersion and surface morphology at the nanoscale. On the other hand, transmission electron microscope (TEM) provides us information on the size, shape, and number of material layers, which vary from low to high resolution. Nonetheless, when SEM (resolving power about 2 nm and maximum magnification about 100,000x) and TEM (resolving power about 0.2 nm and maximum magnification about 1,000,000x) are combined with energy-dispersive X-ray spectroscopy (EDS) detailed information about the metals present in NPs can be obtained [139]. In the case of intracellular NPs synthesis, the localization of synthesized NPs can be determined by the use of SEM and TEM. However, in order to determine the exact size, shape, and crystalline structure of NPs, high-resolution transmission electron microscopy (HR-TEM) is certainly needed. Concerning the surface topography of NPs, the application of an atomic force microscope (AFM) is needed, which can provide three-dimensional information of NPs [33, 231]. UV-Vis spectroscopy oversees the metallic NPs having marked optical characteristics owing to surface plasmon resonance (SPR), preferably in the range of 190 to 1,100 nm [232].

The analysis of striking characteristics can be measured by the interaction of radiations with the metallic NPs, leading to the promotion of electronic transition from the ground state to the higher energy state, which generates a specific SPR band to obtain the size and shape of NPs [233]. Based on this concept, several NPs have demonstrated different absorption spectra for gold, silver, and zinc oxide NPs between 500 and 550 nm, 400 and 450 nm, and 350 and 390 nm, respectively [132, 233–235]. In FTIR spectroscopy, functional groups, which are attached to the NPs, are identified, typically ranging between 4,000 and 400 cm^−1^. While few common functional groups that attach themselves to the NPs include eSHe, eC=Oe, and eNH2e [236, 237]. Brunauer–Emmett–Teller (BET) technique helps determine the specific area of NPs. The behavior of NPs in a liquid environment can be characterized using dynamic light scattering (DLS) and zeta (*ζ*) potential measurements. More specifically, the hydrodynamic diameter, surface charge, and distribution of NPs in liquid and their stability are determined by *ζ*-potential [233].

## 8. Green NPs as an Anti-Bacterial Agent

Antibiotic resistance shown by pathogenic bacteria has increased the necessity to check anti-bacterial potential of metallic NPs. Consequently, it is obligatory to search for novel therapeutic agents for treating multidrug resistant (MDR) pathogens. In this connection, biologically synthesized metallic NPs have attracted many researchers to utilize them as a novel nanomedicine [238–240]. The development of green NPs as anti-bacterial agents has created a new scope in biomedical sciences. Biogenic selenium NPs produced from *Ulvan* extract (*Ulva lactuca*) has been used for producing the mouth rinse that killed oral pathogens (*Streptococcus mutans*, *Staphylococcus aureus*, *Lactobacillus*, and *C. albicans*) at an effective concentration of 100 *μ*g/ml [241]. Polysaccharides-based silver NPs produced from brown macroalgae (*S. cichorioides* and *F. evanescens*) demonstrated a greater zone of inhibition against *Agrobacterium tumefaciens*, as compared to *E. coli* [100]. Silver NPs, green synthesized from the extracts of *S. muticum* exhibited anti-bacterial efficacies by inhibiting the growth of *K. pneumoniae*, *Bacillus subtilis*, *Salmonella typhi*, and *E. coli* [104]. Silver NPs biosynthesized using marine algae (*S. wightii* and *V. pachynema*) affected the growth of *Micrococcus luteus* and *Serratia marcescens* [110]. Silver NPs from red macroalgae *P. hornemannii* have demonstrated the killing of fish pathogens (*Vibrio anguillarum*, *Vibrio harveyii*, *Vibrio alginolyticus*, and *Vibrio parahaemolyticus*) [113]. Green synthesis of silver NPs using *Gelidium* extract demonstrated anti-microbial effects against *E. coli* and *C. albicans*. In addition, the authors have found substantial inhibition of biofilm formation after treatment with silver NPs [114]. In the same context, anti-biofilm effects have been reported by the iron oxide NPs produced from the extracts of three marine macroalgae (*S. vulgare*, *U. fasciata*, and *J. rubens*) [112]. Biogenic production of silver NPs from *C. hornemannii* also exhibited anti-bacterial effects against a range of pathogenic bacterial strains (*Pseudomonas aeruginosa*, *S. aureus*, and *E. coli*) [115].

*Chlorella pyrenoidosa* exhibited a high degree of consistency in the synthesis of silver NPs that actively inhibited the growth of *K. pneumoniae*, *Aeromonas hydrophila*, *Acenetobacter*, and *S. aureus* [242]. Silver NPs produced by the use of extracellular extracts from marine macroalgae (*Caulerpa racemosa*) demonstrated anti-bacterial activities [243]. Moreover, the blue-green alga *Spirulina platensis* also synthesized gold NPs that have effectively killed *B. subtilis* and *S. aureus* [244]. In addition to the anti-bacterial activities, NPs synthesized by macroalgae extracts do have stabilizing effects on cotton fabrics [245]. *Gelidiella acerosa* is a red macroalgae whose extracellular extract produced silver NPs, exhibited fungal growth inhibition [246]. *U. fasciata* exhibited the reduction of silver nitrate salt to silver NPs, which ultimately affected the growth of *Xanthomonas campestris pv. malvacearum* [247]. Aqueous extract of brown macroalgae (*Sargassum longifolium*) resulted in the formation of silver NPs. The synthesized silver NPs acted as a potent anti-fungal agent against pathogenic fungi [84]. Despite the manifold benefits of biogenic NPs, little work has been done on the marine macroalgae especially from the Red Sea of Saudi Arabia. *Galaxaura elongate* (red algae) from the coastal area of Jeddah, Saudi Arabia, has been involved in the synthesis of gold NPs that also demonstrated anti-bacterial effects [248]. Silver NPs synthesized using a red algae (*Laurencia papillosa*) from the coastal area of Jeddah, Saudi Arabia, exhibited bactericidal and anti-fungal effects, indicating its effectiveness as an anti-microbial agent [249].

Silver NPs (13–76 nm) biosynthesized using deep-sea *P. aeruginosa* also demonstrated anti-bacterial efficacies against human pathogens such as *Vibrio cholerae*, *Aeromonas* sp., *E. coli*, and *Corynebacterium* sp. In addition, the NPs effectively hindered the biofilm formation in exposed pathogens (*S. aureus* and *P. aeruginosa*) [250]. *Trichoderma viride*-mediated silver NPs generation showed the killing of human pathogenic bacterial strains (*S. aureus*, *M. luteus*, *S. typhi*, and *E. coli*) at the minimal inhibitory concentrations (MIC) of 80, 65, 35, and 30 *μ*g/ml [251]. The anti-bacterial activity of metallic NPs depends on size and dose, which varies with different strains of pathogens. Similarly, silver NPs synthesized using marine bacteria (*Streptomyces* sp.) showed the anti-bacterial effects against MDR strains (*S. aureus* and *E. coli*) [252]. A possible mechanistic effect of metallic NPs on bacteria can be related to the fact that silver ions may trigger detachment of cytoplasmic membrane from the bacterial cell wall and condense the DNA simultaneously [253]. *Candida* sp. VITDKGB utilized for silver NPs synthesis demonstrated promising anti-bacterial effects against MDR and *K. pneumonia* and *S. aureus* [203]. The differences in anti-bacterial effects have also been related to the cell wall compositions in varying bacterial species. Extracellular synthesis of cadmium sulfide NPs (50–180 nm) using *Enterococcus* sp. increased the zone of inhibition against *E. coli*, *Klebsiella planticola*, *Vibrio* sp., *Serratia nematodiphila*, and *Planomicrobium* sp. [84]. Silver chloride NPs synthesized by green algae (*C. vulgaris*) declined the bacterial survival to 98% and disturbed the normal arrangement of chromosomal DNA in *K. pneumoniae* and *S. aureus* [254]. Compared to chemically synthesized NPs, gold NPs derived from biological sources showed 96.67% greater anti-bacterial activity at 30 *μ*M [255]. Nickel NPs synthesized using the root of *Desmodium gangeticum* demonstrated anti-bacterial activity [256]. Relative to chemically synthesized zinc NPs, the biologically synthesized zinc NPs exhibited excellent anti-bacterial activities against *B. subtilis* ATCC 6633, *Salmonella typhimurium* ATCC 14028, and *M. luteus* ATCC 9341 [257]. The precise anti-bacterial action of NPs is still in its infancy. However, the reported evidences clearly suggest the inhibition of cell membrane architecture, disintegration of proteins and DNA, inhibition of nutrient uptake, oxidation of proteins, inhibition of electron transport chain, and dysfunction of membrane potential. Such effects can also be related to the increased oxidative stress by reactive oxygen species (ROS), which may trigger bacterial cell death [163].

## 9. Application of Green NPs as an Anti-Cancer Agent

The biocompatibility of green NPs has opened a new opportunity to use them as a novel and promising anti-cancer agent. As a matter of fact, the majority of metal-based NPs bio-fabricated using algal sources have been enormously tested for their anti-microbial activity. However, very few studies have been conducted on them to quantify their efficacy as anti-cancer tools. In this line, gold NPs produced from fucoidan of *P. tetrastromatica* significantly reduced the survival of human alveolar (A549) and human liver cancer cell lines between the concentration range of 1–100 *μ*g/ml [103]. Green synthesis of silver NPs using laminaran and alginate isolated from *S. cichorioides* and *F. evanescens* demonstrated proliferation inhibition of rat glioma cells C6 [100]. Gold and silver NPs prepared from the water extracts of marine brown macroalgae (*Saccorhiza polyschides*) exhibited therapeutic potential via immunostimulant and anti-proliferative activity on immune and tumor cells [102]. Sulfated polysaccharide (D-mannose and chitosan) from *Ulva lactuca* entrapped on functionalized graphene oxide NPs have demonstrated targeted killing of human glioblastoma cells (U87), indicating a promising drug delivery system for the treatment of in vitro glioblastoma [258]. Extracellular synthesis of silver NPs by seaweed *C. hornemannii* showed cytotoxic effects in U937 cell lines. In addition, anti-oxidant activity, differential expression of chemokine, cytokines, and hemolytic activity were also reported by the authors [115]. Silver NPs biosynthesized using four different marine macroalgae (*Turbinaria decurrens*, *J. rubens*, *Sargassum cinereum*, and *Caulerpa racemose*) exhibited anti-proliferative effects in human colorectal carcinoma (HCT116) cells. However, no effects were observed in the normal retina cells (RPE1) [259]. Silver and gold NPs synthesized using two different microalgae (*Oscillatoria* sp. and *S. platensis*) were tested on the human colon (CaCo-2) and cervical (HeLa) cancer cells. Both cancer cells showed a significant reduction in their survival after treatment with gold and silver NPs, indicating their prospects as anti-cancer entities [260]. Green algae (*Dictyosphaerium* sp.) mediated extracellular synthesis of gold NPs and novel gold nanoformulations loaded with diosgenin affected the proliferation of colorectal cancer (HCT116) and breast cancer (HCC1954) cells, signified the low concentration efficacy as anti-cancer nanodrugs [118].

*A. vera*-capped hematite nanoparticles (ALE-Fe_2_O_3_NPs) and biofunctionalized CuO NPs significantly declined the survival of MCF-7 cells [148, 149]. Metallic silver and zinc oxide NPs synthesized via microwave-mediated protocol using macroalgae *Gracilaria edulis* displayed the killing of PC3 and normal African monkey kidney (VERO) cell lines [261]. *Olax scandens* leaves used for the production of colloidal silver NPs have significantly declined the proliferation of human breast carcinoma (MCF-7), human lung cancer (A549), mouse melanoma (B16), and colon cancer (COLO 205) cell lines. Gold NPs (14 nm) biosynthesized using red seaweed (*C. officinalis*) induced necrosis in MCF-7 cells at higher concentrations, indicating their anti-cancer efficacies [164]. HepG2 and K562 cells reduced the gold ions into gold NPs and demonstrated the fluorescent behavior in the in vivo self-bioimaging of tumors [262]. *Butea monosperma* leaf extract utilized for the green synthesis of gold and silver NPs exhibited biocompatibility with the normal (ECV-304 and HUVEC) and cancerous (HNGC2, MCF-7, B16F10, and A549) cells. However, when both NPs were loaded with anti-cancer drugs (doxorubicin), MCF-7 and B16F10 proliferation were disturbed, representing their effectiveness as nanomedicine in cancer therapy [263]. Spherical gold and silver NPs, synthesized using marine actinobacteria (*Nocardiopsis* sp.), when exposed to human cervical cancer (HeLa) cells for 24 h have significantly induced cytotoxicity, leading to apoptotic cell death [264]. In the same line, silver NPs synthesized using marine bacteria (*E. coli*) exhibited anti-cancer effects by reducing the viability of HeLa and A549 cells [265]. The cytotoxicity of NPs has been related to the concentrations, interaction time with cells, size of NPs, as well as the type of cancer cells [250, 266–268].

## 10. Other Applications of Biogenic NPs

Apart from the biomedical applications, biogenic gold NPs and palladium nanocrystals have also been utilized for anti-oxidant and catalytic activities, biosensing, and detection of cancer cells [197, 269–273]. Also, the microbially synthesized cadmium sulfide NPs, a semiconductor, exhibited the prospect for its utilization in the fabrication of diodes [204]. The synthesis of manganese oxide microspheres using green algae showed its application as lithium-ion batteries [126]. Silver NPs biosynthesized using the green method exhibited their biocompatibility in normal cells, as well as harbor the fluorescence properties to be used for the localization of drugs [255, 274]. Biogenic silver NPs were used in the fabrication of an optical fiber-based sensor for the detection of H_2_O_2_ in industrial wastes [275]. Bio-iron nanocatalyst produced from a brown macroalgae (*Sargassum polycystum*) revealed its greater efficiency on the recovery of fatty acid methyl esters (FAME) from the whole-cell transesterification of green microalgae (*Dictyococcus* sp. and *Coelastrella* sp.) [276]. One-pot green synthesis of magnetic algal carbon supported flower-like sulfidated nanoscale zerovalent iron (S-nZVI/AC) composite from *Ulva prolifera*. The indicated NPs have been seen as promising water purification material for the effective removal of bromate [277]. Very recently, silver NPs from the extract of marine brown macroalgae (*S. muticum*) have demonstrated insecticidal effects by killing the larvae and adult mosquito strains of India and Saudi Arabia [104]. Biogenic silver NPs produced from polar seaweed *F. gardeneri* demonstrated an outstanding catalytic efficacy by using NaBH_4_ reduction of 4-nitrophenol to 4-aminophenol [108]. Silver NPs synthesized by freshwater green algae (*C. vulgaris*) demonstrated photocatalytic decolorization of methylene blue in a short span of time, indicating the environmental significance for the removal of dye from contaminated water or industrial effluents [278]. Palladium NPs synthesized from the crude extract of *S. cervicorne* via one-pot green facile synthetic method demonstrated a promising catalytic activity to remove harmful azo dyes [111].

## 11. Conclusions and Future Directions

A key fact on the wider acceptability of green synthesized NPs is that this approach overwhelms the use of toxic chemicals for NPs production. Copious evidences implied the application of diverse biological materials (algae, plant extract, bacteria, actinomycetes, fungus, and viruses) as an eco-friendly and efficient way to synthesize NPs. Amongst these, marine macroalgae and microalgae have emerged as an excellent source to conjugate nanotechnology that can lead us to a new horizon of research. A valid reason for such benefits resides in the fact that macroalgae are sources of protein and high content of bioactive compounds such as polysaccharides (fucoidan and sulfated polysaccharides) that play a crucial role in capping and stabilizing the NPs in the intracellular and extracellular approaches. In spite of the fact, large-scale utilization of algal sources as nanobiofactories is still immature. Several aspects act as limiting factors including slow reaction kinetics and low yield of NPs. Distantly, choice of algae, pH, temperature, nonoptimized culture conditions, poor morphological properties of NPs, and colloidal stability (agglomerations) are auxiliary constraints. Future recommendations are to delineate the elusive knowledge on the mechanism of algal NPs, possibly by using large-scale bioreactors to unravel the reaction kinetics, output, and viability of cells. Moreover, a significant amount of research is needed to precisely identify the role of specific biomolecules that act as reducing and capping agents in algae-mediated NPs synthesis. One of the limitations in algal studies is that researchers have mainly focused on the green synthesis of gold and silver NPs. In fact, the potency of algal extracts or cells to produce NPs using metal precursors viz zinc, platinum, palladium, ruthenium, and silicon is still elusive and warrants future studies. Among the other biological sources, plant extracts containing varying types of active compounds (phenols, tannins, terpene, and alkaloids) act as reducing and stabilizing agents. The intracellular presence of nitrate reductase, reductase, and NADPH-dependent reductases in microorganisms plays a fundamental role as reducing agents. Owing to the presence of indicated enzymes, the cell supernatant of microorganisms could also be used to enhance the reaction rate and production yield. Methods for the purification and extraction of synthesized NPs using different biological sources are still elusive. It is also imperative to focus on detailed methodologies that can help purify and isolate green synthesized NPs. Overall, it can be surmised that pairing nano research with distinct biological entities to produce clean and safe NPs may lead us to new horizons of research by producing application-based products. For several decades, algae (macroalgae and microalgae), microorganisms, and plants have been the choice of materials for biofuel production, biorefinery processes, bioremediation, and so on. In spite of these facts, the intrinsic abilities of algal and microbial cells, as well as extracellular extracts of algae, microbes, and plants to reduce metal precursors into metallic NPs, have paved a novel approach to produce biocompatible NPs. Indeed, green synthesized NPs harbor excellent anti-microbial and anti-cancer efficacies, indicating their prospective application as nanotherapeutics after proper testing and evaluations.

## Figures and Tables

**Figure 1:** Schematic diagram exhibiting size comparison of nanoparticles (NPs) typically in the range of 1–100 nm, as compared to the other structures. Created with BioRender.com with publication license.

**Figure 2:** Schematic diagram of two fundamental approaches (top-down and bottom-up) for the synthesis of NPs. Created with BioRender.com with publication license.

**Figure 3:** Application of different biological materials for the biogenic synthesis of NPs Created with BioRender.com with publication license.

**Figure 4:** Illustration showing variations in extracellular matrix (ECMs) of marine macroalgae (brown, red, and green) and differences in their intracellular biological materials. The figures of marine macroalgae ECMs were adopted from the review of Kloareg et al. [89] and redrawn from the work of Deniaud-Bouët and coworkers [90], as well as updated from the following references for brown macroalgae [91–93], red macroalgae [94–96], and green macroalgae [97]. CW Protein (cell wall protein). Created with BioRender.com with publication license.

**Figure 5:** Schematic diagram showing mechanism of intracellular NPs synthesis in algae. Metallic ions get inside the cytoplasm, thereby getting reduced by nitrate reductase enzymes produced from different biochemical reactions. Several biogenic molecules act as capping agents to stabilize finally producing biogenic metallic NPs. However, the extracellular mechanism involves the trapping of metal ions near the cell wall or ECMs, which contain several reducing agents, as well as there is secretion of reducing enzymes and metabolites to the external environment. Altogether, they assist the reduction of metal ions to finally produce capped and stabilized metallic NPs. Created with BioRender.com with publication license.

**Figure 6:** Illustration exhibiting green synthesis of NPs using extracellular extract of macroalgae without heating. Created with BioRender.com with publication license.

**Figure 7:** Schematic representation of metallic NPs synthesis using plant extracts. Image source and credit [177].

**Figure 8:** Summarization of popular methods for characterization of NPs. Created with BioRender.com with publication license.

## Data Availability

The data supporting this review were taken from previously reported studies and data sets, which have been cited.
